# Long noncoding RNA MALAT1 enhances the docetaxel resistance of prostate cancer cells via miR‐145‐5p‐mediated regulation of AKAP12

This article has been retracted.

**DOI:** 10.1111/jcmm.13604

**Published:** 2018-04-06

**Authors:** Dong Xue, Hao Lu, Han‐Yan Xu, Cui‐Xing Zhou, Xiao‐Zhou He

**Affiliations:** ^1^ Department of Urology Third Affiliated Hospital Suzhou University Changzhou Jiangsu China

**Keywords:** *AKAP12*, docetaxel, MALAT1, miR‐145‐5p, prostate cancer

## Abstract

Our present work was aimed to study on the regulatory role of MALAT1/miR‐145‐5p/*AKAP12* axis on docetaxel (DTX) sensitivity of prostate cancer (PCa) cells. The microarray data (GSE33455) to identify differentially expressed lncRNAs and mRNAs in DTX‐resistant PCa cell lines (DU‐145‐DTX and PC‐3‐DTX) was retrieved from the Gene Expression Omnibus (GEO) database. QRT‐PCR analysis was performed to measure MALAT1 expression in DTX‐sensitive and DTX‐resistant tissues/cells. The human DTX‐resistant cell lines DU145‐PTX and PC3‐DTX were established as in vitro cell models, and the expression of MALAT1, miR‐145‐5p and *AKAP12* was manipulated in DTX‐sensitive and DTX‐resistant cells. Cell viability was examined using MTT assay and colony formation methods. Cell apoptosis was assessed by TUNEL staining. Cell migration and invasion was determined by scratch test (wound healing) and Transwell assay, respectively. Dual‐luciferase assay was applied to analyse the target relationship between lncRNA MALAT1 and miR‐145‐5p, as well as between miR‐145‐5p and *AKAP12*. Tumour xenograft study was undertaken to confirm the correlation of MALAT1/miR‐145‐5p/*AKAP12* axis and DTX sensitivity of PCa cells in vivo. In this study, we firstly notified that the MALAT1 expression levels were up‐regulated in clinical DTX‐resistant PCa samples. Overexpressed MALAT1 promoted cell proliferation, migration and invasion but decreased cell apoptosis rate of PCa cells in spite of DTX treatment. We identified miR‐145‐5p as a target of MALAT1. MiR‐145‐5p overexpression in PC3‐DTX led to inhibited cell proliferation, migration and invasion as well as reduced chemoresistance to DTX, which was attenuated by MALAT1. Moreover, we determined that *AKAP12* was a target of miR‐145‐5p, which significantly induced chemoresistance of PCa cells to DTX. Besides, it was proved that MALAT1 promoted tumour cell proliferation and enhanced DTX‐chemoresistance in vivo. There was an lncRNA MALAT1/miR‐145‐5p/*AKAP12* axis involved in DTX resistance of PCa cells and provided a new thought for PCa therapy.

## 1 INTRODUCTION

Ranked as the second lethal malignancy among men in United States, prostate cancer (PCa) is one of the most popular human diseases, with approximately more than 220 000 newly diagnosed cases and 27 000 deaths. Moreover, its occurrence and recurrence rates had been significantly increasing both in developing and developed countries.^1^, ^2^, ^3^, ^4^ Androgen deprivation therapy (ADT) first proposed by Charles Huggins et al on their seminal observations is highly effective in controlling metastatic prostate cancer.^5^ Although ADT is effective for some patients, most patients may develop castration resistance PCa (CRPC).^6^ Docetaxel (DTX) has been subsequently used as a standard treatment for these patients with castration‐resistant prostate cancer (CRPC).^7^ In 2015, 2 trials have been proven to improve survival in men with untreated metastatic prostate cancer through simultaneous addition of DTX and ADT.^8^, ^9^ To date, chemotherapy with DTX has been considered as the primary therapeutic choice. However, emergence of DTX resistance after multiple cycles of therapy usually leads to therapeutic failure. The mechanisms of DTX resistance are quite complex and have not been fully figured out.

Long noncoding RNAs (lncRNAs) are commonly defined as transcripts with more than 200 nucleotides in length. They are frequently dysregulated and play important roles in tumourigenesis and cancer metastasis, acting as oncogenes or tumour suppressors.^10^, ^11^, ^12^, ^13^, ^14^ Emerging studies suggest that lncRNAs are involved in the progression of PCa. PCAT‐1, transcribed from the introns of known genes which correlate with the differentiation degree of PCa, was identified as a prostate‐specific regulator of cell proliferation.^15^ Prostate cancer antigen 3 (PCA3), also known as differential display 3 (DD3), has been thoroughly explored as a PCa‐specific biomarker.^16^ Thus, elucidating the roles of lncRNAs in tumours holds great promise for the prevention, early detection and treatment of tumours. Metastasis associated in lung adenocarcinoma transcript 1 (MALAT1) is located on chromosome 11q13 and contains more than 8000 nucleotides.^14^ It was first discovered by Ji et al as a tumour promoter in non‐small cell lung cancer because of its role of promoting cell metastasis and invasion.^14^ Further studies have confirmed that MALAT1 is overexpressed in human hepatocellular carcinoma, bladder, breast, colorectal, gastric, lung, renal, pancreatic and prostate cancers.^12^, ^17^, ^18^, ^19^, ^20^ It is as an independent prognostic parameter in modulating cell metastasis and epithelial–mesenchymal transition (EMT) process. However, the role of lncRNA MALAT1 in PCa development and chemoresistance is poorly investigated, and new research to disclose the potential mechanism is urgently needed.

MiRNAs are small and nonprotein‐coding RNAs containing 20‐22 nucleotides in length, which negatively modulate genes expression at the post‐transcriptional stage or induce mRNA degradation by binding the 3′ untranslated regions (UTRs) of mRNAs.^21^, ^22^ They play an important role in biological processes^23^ and are broadly involved in tumour proliferation, invasion, angiogenesis and drug resistance.^25^, ^26^, ^27^ MiRNAs such as miR‐148a,^27^ miR‐200c,^28^ miR‐205,^28^ miR‐21^29^ and miR‐34^30^ have been reported to modulate drug resistance of PCa. Recent studies have demonstrated that miR‐145‐5p is down‐regulated in several cancer types, including bladder cancer,^31^ breast cancer,^32^ colon cancer 33 and ovarian cancer,^34^ indicating that it is a tumour‐suppressive miRNA. Meanwhile, miR‐145‐5p was reported to be down‐regulated in PCa tissues and associated with the prognosis of PCa, which potentially served as a biomarker for PCa prognosis.^35^ However, the biological role and action mechanisms of miR‐145‐5p in chemotherapy response of PCa are not fully understood. A recent study in colorectal cancer showed that miR‐145‐5p was associated with oxaliplatin treatment response through regulation of G protein‐coupled receptor 98, leading to chemoresistance.^36^ This study indicated that miR‐145‐5p might be implicated in the modulation of chemoresistance in PCa.

In this study, we uncovered the effect of MALAT1 on the chemosensitivity of PCa cells to DTX. We demonstrated that MALAT1 conferred DTX resistance via *AKAP12*, which was modulated by miR‐145‐5p and related to cell invasiveness and chemoresistance of PCa cells. Our research for the first time confirmed that MALAT1 promoted DTX resistance, providing a potential therapeutic approach for PCa patients with DTX resistance.

## 2 METHODS

### 2.1 Clinical samples

Thirty‐six patients who were pathologically diagnosed with PCa and underwent surgery between March 2013 and December 2015 were recruited from the Third Affiliated Hospital of Suzhou University with informed consents. All the patients acquired standard courses of DTX‐based neoadjuvant chemotherapy, while none of them had received any other therapies, ie radiotherapy, hormone castration and immunotherapy. The characteristics of patients are listed in Table S1. Eighteen samples in resistance group and another eighteen in sensitive group were diagnosed by pathologic examination and separated according to the Response Evaluation Criteria in Solid Tumors (RECIST). During surgery, PCa tissues were frozen in liquid nitrogen at once after resection and stored at −80°C for future use. The experiments were approved by the Ethics Committee of the Third Affiliated Hospital of Suzhou University.

### 2.2 Cell culture and treatment

Human PCa cell lines DU145 and PC3 and Human embryonic kidney cell line HEK‐293T were purchased from BeNa Culture Collection Biological Technology Co., Ltd. (Beijing, China). The cells were cultivated in Dulbecco's Modified Eagle Medium (DMEM; Gibco, Grand Island, NY, USA) with 10% FBS and maintained at an incubator containing 5% CO_2_ at 37°C. Resistant PCa cancer cell lines DU145‐DTX and PC3‐DTX were induced by DTX (Sigma, St. Louis, MO, USA). The definite operations were as follows: resistant cell lines were developed over a period of 6 months by stepwise increased concentrations of docetaxel. Cells were continuously maintained in docetaxel, with treatments beginning at 5 nmol/L. Media containing docetaxel were changed every 2‐3 days. As cells displayed resistance to DTX, surviving cells were cultured and the concentration of DTX was gradually increased to a final dose of 80 nmol/L for DU15‐DTX and 50 nmol/L for PC3‐DTX. The acquired cell resistance to DTX was judged based on decreased cell death and increased cell proliferation. After similar passages, DU145 and PC3 cells were utilized in this study as ageing controls. DU145‐DTX and PC3‐DTX were kept in similar media as DU145 and PC3 except that 5 nmol/L DTX was added in the media for DU145‐DTX and PC3‐DTX.

### 2.3 Bioinformatics analysis

The microarray dataset (GSE33455) of differentially expressed lncRNAs and mRNAs in DTX‐resistant PCa cell lines (DU145‐DTX and PC3‐DTX) was retrieved in the Gene Expression Omnibus (GEO) database (https://www.ncbi.nlm.nih.gov/geo/). Fold change value >2 and *P *<* *.05 was the screening criterion to identify the genes and lncRNAs with differential expression, using the R project for statistical computing. On the other hand, follow‐up data for survival analysis of PCa patients were obtained from The Cancer Genome Atlas (TCGA) database (https://tcga-data.nci.nih.gov/tcga/). The binding sites between MALAT1 and miR‐145‐5p, as well as between miR‐145‐5p and *AKAP12* were predicted using miRcode database (http://www.mircode.org/) and TargetScan 7.1 database (http://www.targetscan.org).

### 2.4 Cell transfection

The plasmids pcDNA3.1‐MALAT1, pcDNA3.1‐*AKAP12*, hsa‐miR‐145‐5p mimics, pcDNA3.1‐shMALAT1, pcDNA3.1‐sh*AKAP12* and negative control (NC) were all provided by GenePharma (Shanghai, China). Before transfection, PCa cells (1 × 10^5^) were cultured until 80% confluence. The vectors and miRNAs were transfected, respectively, into PCa cell lines by Lipofectamine 2000 reagent (Invitrogen, Carlsbad, CA, USA) and cultured corresponding media. Cells transfected with recombinant pcDNA3.1 plasmids were cultured with 1 μg/mL puromycin (Beyotime, Shanghai, China) for 36 hours for selection.

### 2.5 qRT‐PCR

The total RNAs from tissues and cells were extracted using Trizol agent (Takara, Tokyo, Japan). cDNA reverse‐transcribed from quantified RNA by PrimeScript™ RT reagent Kit (Takara) before qRT‐PCR was further used for gene amplification according to the SYBR^®^ Premix Ex Taq™ GC (Takara) protocol on 7500 real‐time PCR system (Applied Biosystems, Foster City, CA, USA). With GAPDH and U6 as the internal references, the relative gene expression was analysed by 2^−▵▵ct^ method, and RNA primers used are listed in Table 1.

**Table 1:** Primer sequences for qRT‐PCR

Compound	Primer name	Sequence
MALAT1	Forward	5′‐GGGTGTTTACGTAGACCAGAACC‐3′
	Reverse	5′‐CTTCCAAAAGCCTTCTGCCTTAG‐3′
NEAT1	Forward	5′‐AGCTGCGTCTATTGAATTGGTAAAGTAA‐3′
	Reverse	5′‐GACAGAAAGATCCCAACGATAAAAATAA‐3′
miR‐145	Forward	5′‐ GTCCAGTTTTCCCAGGAATC‐3′
	Reverse	5′‐AGAACAG‐TATTTCCAGGAAT‐3′
AKAP12	Forward	5′‐ GGAATTCGATGGGCGCCGGGAGCTCCAC‐3′
	Reverse	5′‐ CCGCTCGAGGTCATCTTCGTTGGCCCCTG‐3′
U6	Forward	5′‐CTCGCTTCGGCAGCACATA‐3′
	Reverse	5′‐AACGATTCACGAATTTGCGT‐3′
GAPDH	Forward	5′‐GAAGGTGAAGGTCGGAGTC‐3′
	Reverse	5′‐GAAGATGGTGATGGGATTTC‐3′

### 2.6 Dual‐luciferase assay

The fragment of MALAT1 containing the predicted miR‐145‐5p binding site was amplified by PCR and then subcloned into the XhoI/XbaI sites of pmirGLO Dual‐luciferase miRNA Target Expression Vector (Promega, Madison, WI, USA) to form the reporter vector MALAT1‐wild‐type (pmirGLO‐MALAT1‐wt). To mutate the putative binding site of miR‐145‐5p, the sequence of the putative binding site was replaced and named as MALAT1‐mutated‐type (pmirGLO‐MALAT1‐mt). Similarly, 3′UTR of *AKAP12* was chemically synthesized and inserted into the XhoI/XbaI sites of the pmirGLO Dual‐luciferase miRNA Target Expression Vector (Promega) to form the reporter vector *AKAP12*‐wild‐type (pmirGLO‐*AKAP12*‐wt). *AKAP12*‐mutated‐type was constructed, namely pmirGLO‐*AKAP12*‐mt. HEK‐293T, DU‐145, PC‐3, DU‐145‐DTX and PC‐3‐DTX cells were cotransfected with the recombinant plasmids and miR‐145‐5p or the negative control (scrambles) using Lipofectamine 2000 (Invitrogen). Cells were cultivated in the 96‐well plate and collected after 48 hours transfection. Then, the luciferase activity was measured using the Dual‐Luciferase Reporter Assay System (Promega) through a GloMax™ 96 Microplate Luminometer (Promega). Luciferase data were presented as Firefly luciferase activity normalized to the Renilla luciferase.

### 2.7 Western blot

Protein was extracted from tissues using RIPA buffer containing 1/10 Complete Mini protease inhibitor cocktail (Roche, Basel, Switzerland). The protein content was measured with a BCA Protein Assay kit (Beyotime, Shanghai, China). After denaturing at 95°C for 10 minutes, 50 μg of each protein sample was separated on a 12% SDS‐polyacrylamide gel and then transferred to a polyvinylidenefluoride (PVDF) membrane. After blocking with 5% degrease milk in TBST buffer, the membrane was incubated with mouse monoclonal antibody to AKAP12 (ab49849, 1:200; Abcam, Cambridge, MA, USA) and GAPDH (ab8245, 1:500, Abcam) at 4°C overnight. After washing 3 times with TBST buffer every 15 minutes, the membrane was further incubated with HRP‐labelled goat antimouse IgGs (1:200; Abcam) at 37°C for 1 hour. Finally, the results of Western blot were scanned with Chemical Mp Imaging System (Bio‐Rad, Hercules, CA, USA) and analysed by Gel‐ProAnalyzer (software version 4; UnitedBio, USA). GAPDH was used as a loading control for Western blots.

### 2.8 Immunohistochemistry

Paraffin‐embedded tissues of tumours were sectioned at 4.5 μm thickness. Sections were dewaxed and hydrated before antigens recovery by repeated cooling and heating. They were detected by AKAP12 antibody (1:200, Abcam). Visualization was achieved using diaminobenzidine (DAB) substrate, and sections stained with PBS were regarded as the negative staining control. Colour development was observed using a digital camera (Olympus, Tokyo, Japan) and calculated using Image‐Pro Plus software 6.0 (Media Cybernetics, Silver Spring, MD, USA).

### 2.9 MTT assay

MTT kit (Dojindo, Kumamoto, Japan) was applied to investigate cell proliferation. After transfection, 1 × 10^4^ cells were seeded in a 96‐well plate and cultured overnight. Then, original culture medium was replaced with fresh culture medium supplemented with indicated concentration of DTX. At indicated time, 20 μL MTT (5 mg/mL in PBS) was added in each well for 4 hours and the formazan crystals were dissolved in 150 μL dimethylsulphoxide (DMSO; Sigma‐Aldrich, St Louis, MO, USA). The absorbance was measured at 490 nm on a microplate reader (Molecular Devices, Sunnyvale, CA, USA).

### 2.10 Colony formation assay

Transfected cells were trypsinized and dispensed into individual wells of 6‐well tissue culture dishes with a density of 300 cells per well. Following another 14 days under DTX culture (10 nmol/L), 10% formaldehyde was employed to fix colonies for 10 minutes and 0.5% crystal violet was adopted to stain colonies for 5 minutes. Then, the number of colonies was calculated by ImageJ and images were photographed under a light microscope (Olympus, Tokyo, Japan).

### 2.11 TUNEL staining

TUNEL methods were used to monitor the induction of apoptosis and performed following the guidelines recommended in the In Situ Cell Death Detection Kit (Roche). Briefly, transfected cells were pre‐treated with 10 nmol/L DTX for 24 hours, and then cells in each sample were washed and stained according to the manufacturer's instructions. Positively stained cells were counted with an EVOS FL microscope (Thermo Fisher Scientific, Waltham, MA, USA).

### 2.12 Wound healing assay

Transfected cells (1 × 10^5^ cells per well) were inoculated in a 6‐well plate with 10 nmol/L DTX overnight. Afterwards, 1 μL of pipettes’ spearhead was used to scratch a vertical line in the cell plate. PBS was slowly added into the wells to remove the detached cells. Cells in the wells were cultivated in fresh serum‐free medium at 37°C in an incubator with 5% CO_2_. About 24 hours later, the wells were observed and photographed. Each experiment was conducted for 3 times to obtain the average value.

### 2.13 Transwell assay

After 48 hours transfection, the PC3 and PC3‐DTX cells in every group were collected. Then, each chamber was added with 80 μL of Matrigel (Invitrogen) at a ratio of 1:8. 200 μL of serum‐free DMEM medium with 10 nmol/L DTX was added into the upper chamber with 1 × 10^5^ cells inoculated, while complete culture medium was added into the lower chamber. After 24‐hours incubation, remained cells were wiped away using cotton swabs. The cells attached to the lower surface of membrane were fixed in 4% paraformaldehyde at room temperature for 20 minutes, and 0.1% crystal violet was used for staining for 15 minutes. Five fields were randomly chosen to calculate the cell number under a microscope. Each experiment was conducted for 3 times.

### 2.14 Flow cytometry analysis

Transfected cells of each group were centrifuged at 1000 rpm/min, and fixed with the pre‐cold 70% ethanol at 4°C overnight. After that, PBS solution, 1% BSA solution, 100 μL propidium iodide (PI) and 100 μL RNase A were added in sequence. After 30‐minutes incubation in the dark at 37°C, the distribution of the cell cycle of PCa cells was detected by flow cytometry (BD Bioscience, USA).

### 2.15 Tumour xenograft

For this part of the study, a total of 20 BALB/c nude mice were used and grouped into (1) PC3 group (injected with PC3 cells), (2) PC3‐DTX group (injected with PC3‐DTX cells), (3) PC3‐DTX+MALAT1 group (injected with PC3‐DTX cells with MALAT1 overexpression), (4) PC3‐DTX+sh‐MALAT1 group (injected with PC3‐DTX cells with MALAT1 knockdown), (5) PC3‐DTX+sh‐MALAT1 + mimics group (injected with PC3‐DTX cells with MALAT1 knockdown and miR‐145‐5p), and (6) PC3‐DTX+sh‐MALAT1 + AKAP12 group (injected with PC3‐DTX cells with MALAT1 knockdown and AKAP12 overexpression). 0.2 mL of the above cell suspension that contained 1 × 10^7^ cells were injected into the right axillary fossa of every mouse using microsyringes. At 10 days after injection, an intravenous administration of DTX solution (8 mg/kg) in each mouse was performed every 5 days. Tumour sizes were assessed every 5 days with a digital caliper. The tumour volumes (V) were decided by measuring their length (*l*) and width (*w*) and calculated as follows: *V *= l×*w* ^2^/2. These mice were euthanized, and tumour tissues were weighted after 30 days. Nude mice were purchased from Suzhou Medical Laboratory Animal Center (Suzhou, China) and housed under controlled temperature (28°C) and pathogen‐free conditions at Third Affiliated Hospital of Suzhou University. All procedures were performed aseptically in accordance with the institutional guidelines and approved by the Experimental Animal Ethics Committee of Third Affiliated Hospital of Suzhou University.

### 2.16 Statistical analysis

Each in vitro experiment was conducted 3 times to obtain the average value. GraphPad Prism 6.0 software (GraphPad Software, La Jolla, CA, USA) was employed for data analysis. The differences between 2 groups were analysed through Student's *t* test, multigroups’ difference was analysed by analysis of variance (ANOVA). *P* values of less than .05 were recognized statistically significant.

## 3 RESULTS

### 3.1 LncRNA MALAT1 was overexpressed in human DTX‐resistant PCa

Microarray analysis was applied to recognize differentially expressed lncRNAs in DTX‐sensitive (DU145 and PC3) and DTX‐resistant (DU145‐DTX and PC3‐DTX) PCa cell lines. Among them, MALAT1 (log_2_FC = 1.49, adj.*P*.Val = 1.48E‐06) was significantly up‐regulated in DTX‐resistant PCa cells, predicting it might be effective on drug resistance (Figure 1A,B). To further identify that MALAT1 was involved in modulating DXT sensitivity, the expression levels of MALAT1 and NEAT1 (log_2_FC = 1.18, adj.*P*.Val = 1.59E‐06), 2 lncRNAs that had the most striking difference in expression, were examined by qRT‐PCR in DTX‐sensitive or DTX‐resistant tumour tissues. These results indicated that MALAT1 was significantly up‐regulated in DTX‐resistant tumours tissues (*P *<* *.01, Figure 1C). Therefore, MALAT1 was chosen for the forthcoming experiments. The same results were revealed in cell experiments. MALAT1 expression was significantly increased in PC3‐DTX, about 1.8‐fold higher than its expression in PC3 cells, while MALAT1 expression was overexpressed by about 1.4‐fold in DU145 cells than in DU145‐DTX cells (*P *<* *.01, Figure 1D). As revealed in Figure S1A,B, according to the follow‐up data from TCGA database, the disease‐free survival (DFS) and overall survival (OS) of patients with high MALAT1 expression was significantly lower than patients with low MALAT1 expression (*P *<* *.05). Therefore, we concluded that MALAT1 might involve in regulating DTX sensitivity of PCa.

**Figure 1:** MALAT1 was overexpressed in docetaxel (DTX)‐resistant PCa tissues and cells. A, Volcano plot: LncRNA MALAT1 was analysed by lncRNA‐microarray analysis and selected as a promising lncRNA involved in the chemoresistance of PCa. B, Heat map: LncRNA MALAT1 was overexpressed in DTX‐resistant PCa cells (DU145‐DTX and PC3‐DTX) compared with DTX‐sensitive cells (DU‐145 and PC‐3). C and D, LncRNA MALAT1 was up‐regulated in DTX‐resistant PCa tissues and cells detected by qRT‐PCR, which was consistent with microarray analysis results. NC: negative control. **Compared with the PC3 group, *P *<* *.01; ^##^Compared with the DU145 group, *P *<* *.01

### 3.2 LncRNA MALAT1 enhanced DTX resistance in PCa cells

To research the biological function of MALAT1 on drug resistance of PCa cells, MTT and colony formation assays were applied. We first up‐regulated MALAT1 expression in DU145 (PC3) cells and knocked down the expression of MALAT1 in DU145‐DTX (PC3‐DTX) cells. Then, we performed MTT cell proliferation assay on these cells. The survival rate of DU145/PC3‐DTX was higher than DU145/PC3 cells under different doses of DTX treatment, and the survival rate decreased with gradually increase of DTX (*P *<* *.01, Figure 2A,D). Knockdown of MALAT1 in DU145/PC3‐DTX cells significantly enhanced the inhibition effects of 20 nmol/L DTX (10 nmol/L for PC3‐DTX) (*P *<* *.01, Figure 2B,E). We also performed additional assays to confirm the regulation of cell proliferation by MALAT1. Under the treatment of 10 nmol/L DTX, colony formation of DU145/PC3 cells increased by overexpression of MALAT1 and that of DU145/PC3‐DTX cells was inhibited by knockdown of MALAT1 (*P *<* *.01, Figure 2C,F). Taken together, these data indicated that MALAT1 promoted prostate cell proliferation and enhanced the resistance of PCa cells against DTX.

**Figure 2:** MALAT1 enhanced DTX resistance of PCa. A and B, MTT assay: Cell survival rate of DU145‐DTX was significantly higher than that of DU145 at different dose of DTX. Overexpression of MALAT1 in DU145 cells promoted cell proliferation, but MALAT1 knockdown in DU145‐DTX cells significantly inhibited cell proliferation. C, Colony formation assay: colony formation of DU145 cells was more by overexpression of MALAT1 and that of DU145‐DTX cells was less by knockdown of MALAT1. D and E, MTT assay: Cell survival rate of PC3‐DTX was significantly higher than that of PC3 at different doses of DTX. Overexpression of MALAT1 in PC3 cells promoted PCa cell proliferation, but MALAT1 knockdown in PC3‐DTX cells significantly inhibited cell proliferation. F, Colony formation assay: colony formation of PC3 cells was more by overexpression of MALAT1 and that of PC3‐DTX cells was less by knockdown of MALAT1. NC: negative control. *P <* *.05, *P *<* *.01 **Compared with the control group

### 3.3 LncRNA MALAT1 targeted miR‐145‐5p and repressed its expression

By performing bioinformatics analysis, we notified that there was a promising binding site between MALAT1 and miR‐145‐5p (Figure 3A). Thus, we determined to deeply investigate whether MALAT1 could actually regulate miR‐145‐5p expression. We used dual‐luciferase reporter assay to investigate the interaction between miR‐145‐5p and MALAT1. The dual‐luciferase assay results indicated that miR‐145‐5p mimics observably suppressed the luciferase activity of pmirGLO‐MALAT1‐wt but not pmirGLO‐MALAT1‐mut in the 5 cell lines (*P *<* *.01, Figure 3B–F). To further confirm their regulation, qRT‐PCR demonstrated that expression of miR‐145‐5p in PC3‐DTX cell was markedly lower than that of PC3 cell (*P *<* *.01, Figure 3G). Afterwards, PC3‐DTX cells were transfected for MALAT1 knockdown or MALAT1 overexpression. MALAT1 knockdown significantly restored miR‐145‐5p expression in PC3‐DTX cells, while MALAT1 overexpression significantly reduced miR‐145‐5p level in PC3‐DTX cells (*P *<* *.01, Figure 3H). Therefore, we inferred that there was a MALAT1/miR‐145‐5p axis in PCa cells.

**Figure 3:** MALAT1 directly targeted miR‐145‐5p. A, Schematic diagram showed the sequence alignment between miR‐145‐5p and human MALAT1 lncRNA, with blue letters indicating the mutated seed region. B, The dual‐luciferase assay showed that miR‐145‐5p mimics significantly reduced the luciferase activity of pmirGLO‐MALAT1‐wt but not pmirGLO‐MALAT1‐mut, indicating miR‐145‐5p as a target of MALAT1. **Compared with wt MALAT1 + NC group, *P *<* *.01. C, In DU145 cell line, miR‐145‐5p mimics significantly reduced the luciferase activity of pmirGLO‐MALAT1‐wt but not pmirGLO‐MALAT1‐mut. **Compared with wt MALAT1 + NC group, *P *<* *.01. D, In PC3 cell line, miR‐145‐5p mimics significantly reduced the luciferase activity of pmirGLO‐MALAT1‐wt but not pmirGLO‐MALAT1‐mut. **Compared with wt MALAT1 + NC group, *P *<* *.01. E, In DU145‐DTX cell line, miR‐145‐5p mimics significantly reduced the luciferase activity of pmirGLO‐MALAT1‐wt but not pmirGLO‐MALAT1‐mut. **Compared with wt MALAT1 + NC group, *P *<* *.01. F, In PC3‐DTX cell line, miR‐145‐5p mimics significantly reduced the luciferase activity of pmirGLO‐MALAT1‐wt but not pmirGLO‐MALAT1‐mut. **Compared with wt MALAT1 + NC group, *P *<* *.01. G, The expression of miR‐145‐5p in PC3‐DTX cell line was significantly lower than that of PC3 cell line. **Compared with PC3 group, *P *<* *.01. H, The expression of miR‐145‐5p in PC3‐DTX cells transfected with sh‐MALAT1 was higher than that of MALAT1 overexpression, suggesting miR‐145‐5p was suppressed by MALAT1. QRT‐PCR was used to detect the expression of miR‐145‐5p in PCa cells. NC: negative control. **Compared with NC group, *P *<* *.01

### 3.4 LncRNA MALAT1 targeted miR‐145‐5p to promote DTX resistance of PCa

To ensure the correlation between MALAT1/miR‐145‐5p axis and DTX resistance in PCa cells, we first established cells with different expression of MALAT1 and miR‐145‐5p. As shown in Figure 4A, miR‐145‐5p expression was significantly down‐regulated in MALAT1 overexpressing PC3‐DXT cells and up‐regulated in mimics group, whereas MALAT1 attenuated the miR‐145‐5p supplementation induced by transfection of miR‐145‐5p mimics (*P *<* *.05, Figure 4A). Under the treatment of 10 nM DTX, cell viability in 4 groups was detected. MALAT1 overexpression enhanced the resistance of PC3‐DTX cells to DTX treatment and therefore further promoted cell growth, while miR‐145‐5p mimics significantly impaired cell survival (*P *<* *.05, Figure 4B). MALAT1 overexpression neutralized the inhibitory effects of miR‐145‐5p (*P *<* *.05, Figure 4B). TUNEL assay to assess the apoptosis rate confirmed that MALAT1 inhibited apoptosis of PC3‐DTX cells, which was restored by miR‐145‐5p overexpression (*P *<* *.01, Figure 4C). The percentage of cells arrested in G2/M phase decreased significantly in PC3‐DXT cells with MALAT1 overexpression, while the percentage of cells arrested in G2/M phase increased with miR‐145‐5p overexpression (*P *<* *.01, Figure 4D). These results demonstrated that MALAT1 in PC3‐DXT cells could alleviate DTX‐induced cell cycle arrest by sponging miR‐145‐5p. Meanwhile, under the treatment of DTX, MALAT1 overexpression significantly rescued cell‐migratory and cell‐invasive capacity in PC3‐DTX cells, whereas miR‐145‐5p further impaired PC3‐DTX migratory and invasive capacity. The cotransfection of MALAT1 and miR‐145‐5p mimics did not change migratory and invasive capacity compared with NC (*P *<* *.01, Figure 4E,F). Patients with high miR‐145‐5p levels displayed observably higher rate of DFS and OS compared with those with low miR‐145‐5p levels (Figure S1C,D, *P *<* *.05). Taken together, these data indicated that MALAT1/miR‐145‐5p axis could modulate chemotherapy sensitivity of PCa cells.

**Figure 4:** MALAT1 sponged miR‐145‐5p to promote DTX resistance in PCa. A, The miR‐145‐5p expression was significantly down‐regulated after MALAT1 was overexpressed in PC3‐DXT cells, whereas it was alleviated by miR‐145‐5p mimics. B, MTT results showed that MALAT1 overexpression increased the resistance of PC3‐DTX cells to DTX and promoted cell growth under the treatment of 10 nmol/L DTX, while transfection with miR‐145‐5p mimics significantly inhibited cell proliferation. No significant change was observed in PC3‐DXT with MALAT1 and miR‐145‐5p co‐overexpression. C, TUNEL assays revealed that MALAT1 inhibited DTX‐induced apoptosis of PC3‐DTX cells, and miR‐145‐5p overexpression promoted cell apoptosis. No significant cell apoptosis was observed in cells with simultaneous overexpression of MALAT and miR‐145‐5p. D, Flow cytometry results revealed that miR‐145‐5p overexpression enhanced DTX‐induced G2/M cell cycle arrest, which was alleviated by MALAT1. No significant difference was observed in cells with simultaneous overexpression of MALAT and miR‐145‐5p. E, Wound healing assay: MALAT1 promoted the migration of PC3‐DTX cells after the treatment of DTX, while miR‐145‐5p suppressed the migration. The effect of MALAT1 was attenuated by miR‐145‐5p. Bar: 200 μm. F, Transwell assay: MALAT1 significantly rescued cell‐invasive capacity in PC3‐DTX cells under the treatment of DTX, whereas miR‐145‐5p impaired the invasive capacity of PC3‐DTX. Cotransfected with MALAT1 and miR‐145‐5p mimics, invasive capacity was not significantly changed compared with NC group. Bar: 50 μm. NC: negative control. *Compared with control group, *P *<* *.05; **Compared with NC group, *P *<* *.01

### 3.5 *AKAP12* was overexpressed and targeted by miR‐145‐5p in DTX‐resistant PCa cells

Microarray analysis was applied to screen out differentially expressed mRNAs in PC3 and PC3‐DTX PCa cell lines. To find out downstream targets of miR‐145‐5p involved in chemoresistance of PCa cells, we searched the target genes regulated by miR‐145‐5p on miRbase (http://www.mirbase.org/) and miRanda (http://www.microrna.org/). *AKAP12* was observed up‐regulated in DTX‐resistant PCa cells by microarray analysis (Figure 5A,B), and the results were confirmed in DTX‐sensitive and DTX‐resistant tissues by immunohistochemical method (Figure 5C) and Western blot (Figure 5D). Meanwhile, *AKAP12* mRNA level was significantly high in PC3‐DTX cells in comparison with PC3 cells (*P *<* *.05, Figure 5E). Therefore, we decided to further investigate whether miR‐145‐5p could regulate *AKAP12* expression in PCa cells. Their putative binding relationship was presented in Figure 5F. Dual‐luciferase reporter assay was also used to determine the relationship between miR‐145‐5p and *AKAP12*. These results suggested that miR‐145‐5p mimics suppressed the luciferase activity of *AKAP12*‐wt but not *AKAP12*‐mut (*P *<* *.01, Figure 5G‐K), suggesting that *AKAP12* expression was directly inhibited by miR‐145‐5p. TCGA analysis illustrated that DFS and OS of patients with high *AKAP12* levels was significantly lower than patients with low *AKAP12* levels (Figure S1E,F, *P *<* *.05), indicating the prognostic value of *AKAP12* in clinical application for PCa.

**Figure 5:** *AKAP12* was overexpressed and targeted by miR‐145‐5p in DTX‐resistant PCa. A, *AKAP12* was highly expressed in DTX‐resistant PCa cells analysed by mRNA microarray. The results were presented by volcano plot. B, Heat map: *AKAP12* was overexpressed in DTX‐resistant PCa cells (PC3‐DTX) compared with DTX‐sensitive cells (PC‐3). C, The protein level of *AKAP12* was significantly up‐regulated in DTX‐resistant tumour tissues. D, The high expression level of AKAP12 was verified by Western blot. E, The mRNA level of *AKAP12* was significantly overexpressed in DTX‐resistant PCa cells qualified by qRT‐PCR. F, The putative binding site between *AKAP12* and miR‐145‐5p was predicted by TargetScan. G‐K, The dual‐luciferase assay showed that miR‐145‐5p mimics significantly reduced the luciferase activity of *AKAP12*‐wt but not *AKAP12*‐mut, suggesting *AKAP12* directly targeted by miR‐145‐5p in HEK293T (G), DU145 (H), PC3 (I), DU145‐DTX (J) and PC3‐DTX (K) cell lines. NC: negative control. **Compared with wt AKAP12 + NC group, *P *<* *.01. *Compared with control group, *P *<* *.05. **Compared with control group, *P *<* *.01

### 3.6 MiR‐145‐5p suppressed *AKAP12* to reduce DTX resistance of PCa

To test the potential function of miR‐145‐5p/*AKAP12* in resistance of PCa cells to DTX, we first manipulated the expression of miR‐145‐5p and *AKAP12* in PC3‐DTX cells. The expression of *AKAP12* was reduced with miR‐145‐5p overexpression (*P *<* *.01, Figure 6A). The effects of *AKAP12* overexpression, miR‐145‐5p overexpression or simultaneous overexpression of *AKAP12* and miR‐145‐5p on the proliferation of PC3‐DTX cells with 10 nmol/L DTX were determined using MTT assay. The forced overexpression of miR‐145‐5p increased the sensitivity to DTX of cells, while the forced overexpression of *AKAP12* functioned oppositely, including reduced TUNEL positive cells, alleviated G2/M arrest, increased migration and invasion ability under the treatment of DTX compared with in NC group (*P *<* *.01, Figure 6B‐F). The enhanced resistance to DTX induced by *AKAP12* overexpression was attenuated by miR‐145‐5p mimics. These data suggested that miR‐145‐5p played an inhibitory role in DTX resistance of PCa through inhibiting *AKAP12*.

**Figure 6:** miR‐145‐5p suppressed *AKAP12* to reduce DTX resistance of PCa. A, *AKAP12* expression was significantly down‐regulated after miR‐145‐5p was overexpressed in PC3‐DXT cells. B, MTT assay: Increased expression of *AKAP12* enforced resistance to DTX and promoted cell proliferation, but increased expression of miR‐145‐5p enforced sensitivity to DTX at the dose of 10 nmol/L DTX. No significant change was observed in miR‐145‐5p and *AKAP12* co‐overexpression group. C, TUNEL assay: *AKAP12* enhanced the resistance to DTX‐induced apoptosis, but miR‐145‐5p induced the apoptosis of DTX‐resistant cells. No significant change was observed in miR‐145‐5p and *AKAP12* co‐overexpression group. Bar: 50 μm. D, Flow cytometry results revealed that *AKAP12* impaired the DTX‐induced G2/M arrest of PC3‐DTX cells that was enhanced in miR‐245‐5p group. No significant difference was observed in *AKAP12* and miR‐145‐5p simultaneously overexpression group. E, Wound healing assay: *AKAP12* induced the migration of chemo‐resistant PCa cells, while miR‐145‐5p inhibited the migration of PC3‐DTX, which was attenuated by *AKAP12*. Bar: 200 μm. F, Transwell assay: *AKAP12* significantly recovered the invasive capacity of PC3‐DTX cells under the treatment of 10 nmol/L DTX, whereas miR‐145‐5p impaired PC3‐DTX invasive capacity. Cotransfected with MALAT1 and miR‐145‐5p mimics, invasive capacity was not significantly changed compared with NC. Bar: 50 μm. NC: negative control. *Compared with control group, *P *<* *.05. **Compared with NC group, *P *<* *.01

### 3.7 LncRNA MALAT1 promoted PCa cell proliferation in vivo

To further validate the effects of MALAT1 on chemoresistance of PCa cells to DTX in vivo, PC3 cells, PC3‐DTX cells, MALAT1 overexpressed PC3‐DTX cells, MALAT1 knockdown PC3‐DTX cells, MALAT1 knockdown and miR‐145‐5p suppression PC3‐DTX cells as well as MALAT1 knockdown and AKAP12 overexpression PC3‐DTX cells were injected to mice to build in vivo models. All mice underwent an administration of DTX every 5 days, and tumour sizes were recorded during the experiment. Compared with the tumour growth in PC3 group, tumour size in PC3‐DTX increased rapidly. Strongly enhanced tumourigenesis was observed in MALAT1 overexpressed PC3‐DTX cells, while down‐regulation of MALAT1 in PC3‐DTX cells inhibited the tumour formation significantly. At thirty days after injection, tumours were isolated and weighed. Tumour weight in PC3‐DTX with up‐regulation of MALAT1 was heaviest, while in PC3‐DTX knocked down of MALAT1 the tumour weight was lighter compared with in PC3‐DTX group. In addition, the simultaneous modulation of MALAT1 and miR‐145‐5p or AKAP12 led to no significant difference from PC3‐DTX group in terms of tumour growth and weight (*P *<* *.01, Figure 7A‐C). To confirm the signal transduction pathway as mentioned above in vivo, we assessed the expression of MALAT1, miR‐145‐5p and *AKAP12*. QRT‐PCR method confirmed that the MALAT1 and *AKAP12* expression levels were significantly higher, whereas miR‐145‐5p expression level was lower in PC3‐DTX and PC3‐DTX+MALAT1 group compared to PC3 group. Similarly, the expression of MALAT1 and *AKAP12* in PC3‐DTX+shMALAT1 was significantly lower than PC3‐DTX group. The levels of MALAT1 and *AKAP12* were not significantly different from PC3‐DTX group but significantly higher than those of PC3 group. On the other hand, the level of miR‐145‐5p was significantly lower in PC3‐DTX+shMALAT1 + inhibitor group and significantly higher in PC3‐DTX+shMALAT1 + AKAP12 group than in PC3 group (Figure 7D). Besides, Western blot displayed the same trend in AKAP12 expression among different groups (*P *<* *.01, Figure 7E). Thus, these data complemented the studies of the functions of MALAT1 in vitro, suggesting that MALAT1 was capable of promoting the expression of *AKAP12* by down‐regulating miR‐145‐5p to promote DTX resistance.

**Figure 7:** MALAT1 promoted PCa cells proliferation in nude mice. A, Tumours were excised and photographed 30 days after tumour cells inoculation. B and C, Tumour volumes and weight were detected. Xenograft study illustrated that the overexpression of MALAT1 promoted tumour growth but MALAT1 knockdown inhibited tumour growth. In addition, the simultaneous modulation of MALAT1 and miR‐145‐5p or *AKAP12* led to no significant difference from PC3‐DTX group in terms of tumour growth and weight. D, Real‐time PCR analysis demonstrated that the expression of MALAT1 and *AKAP12* significantly increased, while miR‐145‐5p expression decreased in DTX plus MALAT1‐treated tumours compared to their counterparts, completely opposite results were reflected by DTX plus sh‐MALAT1‐treated tumours group. The simultaneous modulation of miR‐145‐5p and AKAP12 reversed the effects of MALAT1 knockdown. E, Western blot was utilized for detecting the AKAP12 protein expression in isolated tumours. NC: negative control. *P <* *.05, **P <* *.01, Compared with PC3 group. ^##^ *P *<* *.01, compared with PC3‐DTX group

## 4 DISCUSSION

In this study, we firstly found that lncRNA MALAT1 was overexpressed in DTX‐resistant PCa cells and revealed its effect on mediating DTX resistance of PCa. Overexpressed MALAT1 in PCa cells enhanced chemoresistance of PCa to DTX, induced cell proliferation, migration and invasiveness, as well as inhibited cell apoptosis. Knockdown of MALAT1 in DTX‐resistant PCa cells up‐regulated miR‐145‐5p as well as suppressed *AKAP12* expression, further inhibited cell viability and induced apoptosis. Our findings suggested there was a MALAT1/miR‐145‐5p axis in modulating chemoresistance of PCa cells to DTX.

Numerous lncRNAs have been reported to affect the drug resistance of cancers, indicating lncRNAs can serve as biomarkers/targets of drug resistance in cancer progression.^37^, ^38^, ^39^ LncRNA MALAT1 was first recognized as a marker for metastasis development in the early stages of lung adenocarcinoma^14^ and recently in PCa.^40^ It has been shown to play an important role in multiple cancers via various mechanisms, such as acting as miRNA sponges, enhancing EMT and stimulating apoptosis or autophagy.^12^, ^17^, ^18^, ^19^, ^20^ Recently, MALAT1 has been confirmed to induce chemoresistance to oxaliplatin of colorectal cancer by promoting *EZH2* 41 and regulate multidrug resistance of hepatocellular carcinoma cells by sponging miR‐216b to modulate the expression of *HIF‐2*α that is related to autophagy pathway.^42^ A previous study has shown that MALAT1 is overexpressed in PCa and is a biomarker of poor prognosis,^40^ indicting it may be involved in modulating chemoresistance of PCa. In our study, we identified MALAT1 level was significantly higher in DTX‐resistant tumour tissues and cells than in DTX‐sensitive tumour tissues and cells. Subsequently, forced overexpression of MALAT1 enhanced the chemoresistance of PCa to DTX, further induced cell growth and aggression as well as inhibited cell apoptosis.

MiRNAs have been reported to play important roles in tumourigenesis, metastasis and multidrug resistance (including paclitaxel, DTX and enzalutamide) in prostate cancer.^2^, ^43^, ^44^, ^45^ MiR‐145 has been found to be sponged by lncRNA‐ROR and therefore causes chemoresistance and EMT phenotypes of DTX‐resistant lung adenocarcinoma cells.^46^ Another study proposed that the inhibition of miR‐145‐5p reversed drug resistance to oxaliplatin in colorectal cancer cell line by regulating the expression of drug‐resistant proteins G protein‐coupled receptor 98.^36^ In addition, miR‐145‐5p was reported to sensitize gallbladder cancer to cisplatin by regulating multidrug resistance associated protein 1.^47^ There are no studies that have been published on the effects of miR‐145 on drug resistance of PCa. Thus, we found that MALAT1 could directly suppress miR‐145‐5p expression, leading to the chemoresistance of PCa cells to DTX. These results indicated that the forced expression of miR‐145‐5p in PCa cells might cause chemosensitivity of PCa cells to DTX.

The underlying mechanism about the effects of miR‐145‐5p on chemoresistance was investigated in our study as well. *AKAP12* was confirmed as a promising target of miR‐145‐5p. A previous study revealed that *AKAP12* promoted cell invasiveness and chemoresistance,^48^ implying its role in enhancing chemoresistance. In this study, we discovered that the expression of *AKAP12* was enhanced by miR‐145‐5p deficiency, which therefore promoted chemoresistance of PCa cells to DTX.

There are still some limitations in our study. Detailed mechanisms of MALAT1/miR‐145‐5p/*AKAP12* axis regulating chemoresistance of PCa cell are still elusive. MALAT1 as a novel biomarker and target for overcoming chemotherapy resistance remains to be further investigated in clinical. In addition, the follow‐up data of these thirty‐six patients are not available at this stage, making the result of our research less convinced.

Collectively, the DTX resistance of PCa cells can be regulated by MALAT1/miR‐145‐5p/*AKAP12* axis. The modulation of this axis also contributes to the inhibitory efficiency of DTX on tumourigenesis in vivo. Our findings may contribute to the comprehension of DTX resistance of PCa, therefore helping with effective treatment for PCa.

## 5 CONCLUSION

In conclusion, the overexpression of MALAT1 contributes to the DTX resistance of PCa cells by sponging miR‐145‐5p and subsequently increasing *AKAP12* level. MiR‐145‐5p was suppressed by MALAT1 in DTX‐resistant PCa cells and might work as a tumour suppressor in PCa progression by targeting *AKAP12*. Briefly, a MALAT1/miR‐145‐5p/*AKAP12* axis was demonstrated to regulate chemosensitivity of PCa cells to DTX. On account of the crucial role of MALAT1 and miR‐145‐5p in PCa drug resistance, it holds great expectation as a potential therapeutic target for PCa resistance to DTX.

## RESEARCH INVOLVING HUMAN PARTICIPANTS AND/OR ANIMALS

All procedures performed in studies involving human participants were in accordance with the ethical standards of Third Affiliated Hospital, Suzhou University.

## INFORMED CONSENT

Approval was obtained from the ethic committee of Third Affiliated Hospital, Suzhou University.

## CONFLICT OF INTEREST

No conflict of interest exits in the submission of this manuscript, and this manuscript has been approved by all authors for publication.

## AUTHOR CONTRIBUTION

Substantial contributions to research design, or the acquisition, analysis or interpretation of data: Hao Lu and Han‐Yan Xu; Drafting the paper or revising it critically: Dong Xue and Cui‐Xing Zhou; Approval of the submitted and final versions: Xiao‐Zhou He.
